# Body Mass Index Showed No Impact on the Outcome of In Vitro Fertilization in Progestin-Primed Ovarian Stimulation Protocol

**DOI:** 10.1155/2021/9979972

**Published:** 2021-09-17

**Authors:** Zhe Yang, Xuehan Zhao, Xue Hu, Xiangyang Ou, Tailang Yin, Jing Yang, Gengxiang Wu

**Affiliations:** ^1^Reproductive Medical Centre, Renmin Hospital of Wuhan University, Jiefang Road 238, Huanghelou Street, Wuhan 430060, Hubei Province, China; ^2^Department of Human Reproductive Medicine, Beijing Obstetrics and Gynecology Hospital, Capital Medical University, Yaojiayuan Road 251, Chaoyang District, Beijing 100026, China; ^3^Reproductive Medicine Center, Taihe Hospital, Renmin South Road 32, Maojian District, Shiyan City, Shiyan 442000, Hubei Province, China

## Abstract

**Purpose:**

To assess whether body mass index (BMI) affects the outcome of in vitro fertilization (IVF) in progestin-primed ovarian stimulation (PPOS) protocol.

**Methods:**

A retrospective study was conducted in the Reproductive Medicine Center, Renmin Hospital of Wuhan University, from June 2016 to June 2017. 636 infertile women who received PPOS protocol in IVF treatment were divided into three groups according to BMI. The data of basic characteristics, embryological outcomes, and cycle characteristics of controlled ovarian stimulation of different groups were collected and studied. *Result(s)*. There was no significant difference in almost all the basic characteristics, embryological outcomes of controlled ovarian stimulation, and cycle characteristics of controlled ovarian stimulation among the three groups. There was a tendency that the duration of infertility was decreased with the increase of patients' weight, although there was no significant difference (*P*=0.051). However, overweight patients had a higher fertilization rate than normal weight patients and underweight patients (70.3 vs. 67.7 vs. 66.8, *P*=0.008), but two-pronuclei (2PN) fertilization rate and cleavage rate showed no significant difference among the three groups. *Conclusion(s)*. BMI showed no impact on the outcome of the ovarian stimulation outcome in PPOS protocol. PPOS protocol may benefit overweight patients, for it attains the same effect with normal patients and requires no increase in gonadotropin (Gn) dose and Gn duration.

## 1. Introduction

Progestin-primed ovarian stimulation (PPOS) protocol is a new ovarian stimulation regimen based on a freeze-all strategy that uses progestin as an alternative to a gonadotropin-releasing hormone (GnRH) analog for suppressing a premature luteinizing hormone (LH) surge during the follicular phase [1]. PPOS can effectively prevent the activation and transmission phases of 17*β*-estradiol (E2) induced LH surges and thus serves as an alternative to conventional treatment with GnRH analogs [2]. This new regimen of ovarian stimulation has been proved to availably prevent a premature LH surge and does not compromise oocyte competence in cycles followed by embryo cryopreservation. It has been widely used in patients receiving in vitro fertilization (IVF) since 2016 and showed good IVF outcomes [3, 4]. Indeed, a PPOS protocol may be considered more “user friendly” for the patients in view of its advantage of fewer injections than a conventional protocol [5]. In this study, we showed the efficacy of PPOS protocol in various patients and validated its safety in embryonic morphology. Patients can benefit from this protocol for its effectiveness in preventing early LH surges and getting satisfactory pregnancy outcomes under much more simple and economic administrations.

Previous studies revealed that various factors may affect and predict clinical outcomes of IVF including age, weight, basal serum follicle-stimulating hormone (FSH) concentration, the number of antral follicles, the newly detected anti-Mullerian hormone (AMH), and so on [6, 7]. According to these researches mentioned above, patients' weight has shown a profound impact on ovarian responses, and it may be related to individual variations. For instance, overweight and underweight patients may suffer a high cycle cancellation rate, poor ovarian response, and a low clinical pregnancy rate and live birth rate after IVF treatments [8–12].

Body mass index (BMI) is usually used as an important factor to calculate the dosage of gonadotropins during the controlled ovarian stimulation (COH). The available evidence about the effects of BMI on the outcome of assisted reproductive technology (ART) is conflicting [13]. Most studies agree that the increase in BMI is related to the increase amounts of gonadotropins used in the process of COH [14], but others found that there is no significant difference in the gonadotropin doses between different BMI groups [15]. Carrell et al. reported that BMI is inversely related to intrafollicular human chorionic gonadotropin (hCG) concentrations, embryo quality, and IVF outcome [16], while some other studies found that BMI has no effect on the final IVF pregnancy outcomes [9, 15, 17]. However, the studies mentioned above were all focused on the traditional COH protocols, such as GnRH agonist (GnRH-a) and GnRH antagonist (GnRH-an) protocols, and there are few studies about PPOS protocol until now.

In conclusion, the impact of BMI on the outcome of PPOS has not yet been evaluated. Therefore, a retrospective study was performed to preliminarily investigate the influence of BMI on PPOS outcome and to provide data for future clinical practice in COH.

## 2. Patients and Methods

### 2.1. Study Population

This retrospective study involved 636 infertile women who received PPOS protocol (details as follows) during IVF or intracytoplasmic sperm injection (ICSI) treatment in the Reproductive Medicine Center, Renmin Hospital of Wuhan University, from June 2016 to June 2017. The participants recruited in this study were women who were between 23 and 48 years old, and patients who had chromosomal abnormalities were excluded. According to a previous study about the Chinese BMI and its related risk factors [18], patients were divided into three subgroups according to BMI: BMI < 18.5 Kg/m^2^ was assigned to underweight group, 18.5 ≤ BMI < 24 Kg/m^2^ was assigned to normal weight group, and BMI ≥ 24 Kg/m^2^ was assigned to overweight group.

This study was approved by the ethical committee of Renmin Hospital of Wuhan University, and informed written consent was obtained from all patients (Ethics Number: WDRY2016-K017).

### 2.2. Controlled Ovarian Stimulation

At the beginning of this process, patients were administrated 10 mg/d medroxyprogesterone acetate (MPA, Beijing ZhongXin Pharmaceutical, China), and they received a daily injection of 150 to 300 IU human menopausal gonadotrophin (hMG, Livzon Pharmaceutical Group Co., China) from menstrual cycle day 2 or 3 on the day of hCG administration. For the purpose of height measurement and clinical requirement, transvaginal ultrasound and serum E2 concentrations were used to monitor the IVF cycle every 2 to 3 days. After testing of the index of E2 concentrations and ovarian responses, the dose of HMG was adjusted according to these indexes. Final oocyte maturation was triggered by 10000 IU hCG (Livzon Pharmaceutical Group Co., China) when three or more dominant follicles reached 18 mm in diameter. Oocyte retrieval was performed 36 hours later under the guidance of transvaginal ultrasound, and all follicles greater than 10 mm in diameter were retrieved.

### 2.3. IVF Procedures and Embryo Freezing

The procedures of IVF/ICSI, embryo culture, and embryo freezing have previously been described by the colleagues in the same department [19]. Fertilization results were assessed 18 h after IVF/ICSI for the appearance of two distinct pronuclei and two polar bodies. 48 h (day 2) and 72 h (day 3) after oocyte retrieval, the embryo morphology was observed and graded. The grading criteria for the embryos were as follows: grade I (equal size of blastomeres, free of fragmentation), grade II (unequal size of blastomere, fragmentations <20%), grade III (unequal size of blastomere, fragmentations 20%–50%), and grade IV (unequal size of blastomere, fragmentations >50%). Finally, on the 3rd day, all high-quality embryos were cryopreserved, and patients were advised to transfer thawed embryos three months later. The definition of 3 top quality of embryos on day 3 is grade 1–2 embryos at 72 h after oocyte retrieval.

### 2.4. Data Collection

The basic characteristics such as the age (years), duration of infertility (years), previous pregnancy (%), previous IVF failures, cause of infertility (%) (including tubal factor, endometriosis, dysfunction of ovulation, male factor, and combined factor), antral follicle counts, basal FSH concentration (mIU/mL), basal LH concentration (mIU/mL), and basal E2 concentration (pg/ml) were recorded. The cycle characteristics of controlled ovarian stimulation such as the Gn dose (IU), Gn duration (days), >10 mm follicles on HCG day (*n*), >14 mm follicles on HCG day (*n*), E2 concentration on HCG day (pg/ml), endometrium thickness on hCG day (mm), oocytes retrieved (*n*), fertilized eggs (*n*), cleaved embryos (*n*), fertilization rate (%), cleavage rate (%), 2PN fertilization rate (%), 2PN cleavage rate (%), cancellation rate of the cycle (%), and top quality of embryos of day 3 (*n*) were calculated, respectively.

### 2.5. Hormone Measurement

The serum basal levels of FSH, LH, and E2 on the 2nd day of the menstrual cycle and E2 on HCG day were also detected. Hormone levels were measured by the chemiluminescence method (Simens, ADVIA Centaur System, USA).

### 2.6. Statistical Analysis

Continuous data were presented as mean ± standard deviation (SD) and tested using the ANOVA test. Noncontinuous data were presented as a percentage (%) and tested using the chi-Square test. *P* < 0.05 was considered statistically significant. Statistical analysis was performed using the IBM SPSS Statistic 23 (IBM, Armonk, NY, USA).

## 3. Results

### 3.1. Patients' Characteristics

There was no significant difference in almost all the basic characteristics between the three groups, including age, previous pregnancy rate, antral follicle counts, basal hormone concentration, and the causes of infertility. There was a tendency that the duration of infertility was decreased by the patients' weight, although there was no significant difference (*P*=0.051) (Table 1).

### 3.2. Ovarian Stimulation and Embryologic Characteristics

During the ovulation stimulation processes, not only the gonadotropins (Gn) dose and Gn duration but also the follicles with diameter greater than 10 mm or 14 mm, E2 concentration, and endometrium thickness on HCG day showed no statistically significant differences among different weight groups. There was no significance in the number of oocyte retrieved and top quality of embryos on day 3. However, overweight patients had a higher fertilization rate than normal weight patients and underweight patients (70.3 vs. 67.7 vs. 66.8, *P*=0.008), but two-pronuclei (2PN) fertilization rate, cleavage rate, and the cancellation rate of the cycle showed no significant difference among the three groups (Table 2).

## 4. Discussion

With the utilization of GnRH-a and GnRH-an protocols in controlled ovarian stimulation, the outcome of clinical ovarian stimulation treatment has been obviously promoted. However, there are still some patients suffering from cycle cancelled due to early surges of LH and lack of oocytes, especially for the patients who have a poor ovarian reserve. Kuang et al. firstly reported that using HMG and letrozole in luteal phase can effectively reduce the early surge of LH and can have an optimal pregnancy in the following frozen embryo transfer (FET) treatment for patients who have normal ovarian reserve [4]. Furthermore, they applied this method, which was termed as PPOS protocol later on, artificially creating a high level of progesterone in follicular phase by oral progesterone feeding, and acquired great outcomes in ovarian stimulation and pregnancy [1, 20].

The critical point of PPOS protocol is the continuous high level of progesterone, which could block the positive feedback of the estrogen and can effectively restrain the emergence of LH surges. PPOS protocol has been verified functional in patients with polycystic ovarian syndrome (PCOS) [21] or poor ovarian reserve [22] for its success in the reduction of LH surges. Kuang et al. reported that PPOS protocol in combination with embryo cryopreservation as an ovarian stimulation regimen was as effective as GnRHa long protocol during COH under different endocrine mechanisms [23]. In view of the amount of the benefits for the patients and the fast developments in FET technology, which ensured the security and interests of patients, such as the reduction in administration time and the relief of patients' economic burden, PPOS protocol has become an optimal protocol in patients undergoing IVF treatments. It has been a preferred solution in many Chinese IVF centers for patients with poor ovarian reserve nowadays. As all embryos should be frozen in this protocol, it is also used in these high responders to prevent ovarian hyperstimulation syndrome (OHSS) in our center.

Clinical observations over the effects of BMI on the ovarian stimulation and pregnancy outcome in other protocols are still controversial. In some studies, scholars came to the conclusion that BMI had no effect on the final IVF pregnancy outcome [9, 17], while the others observed oppositely [8, 10] that increasing BMI did not adversely affect the outcome of IVF in nonobese endometriosis patients [15]. Nevertheless, it was acknowledged that overweight patients require a high dose of Gn [9, 17], a long duration of treatment period [9, 10], a lower estradiol concentration peak [8, 9], even a reduction in oocyte retrieved [17], and an increase in cycle cancellation [10, 17]; despite lack of evidence due to the small number of patients, underweight patients tend to have less embryos portable as some studies mentioned [12]. According to the above conclusion, high-weight patients and low-weight patients have their own advantages and disadvantages which may cause BMI to have no impact on the outcome of in vitro fertilization in progestin-primed ovarian stimulation protocol. Furthermore, our results showed that BMI affects neither the Gn dose and duration nor the oocyte retrieved and top quality of embryos on day 3, which may reveal that BMI may not affect the ovarian stimulation outcome in PPOS protocol.

What is interesting is that the current study showed that the fertilization rate in the overweight group was higher than that of the normal and underweight patients, which pointed out that obesity may affect the fertilization process, while 2PN fertilization rate and cleavage rate showed no significant difference among the three groups. A probable explanation for this elevation could be the higher percentage of PCOS patients in the overweight group, who were detected to have a higher rate of abnormal fertilization rate, which was in agreement with a previous study reported by Beydoun et al. [24]. Usually, obesity may be responsible for the Gn resistance during ovarian stimulation according to the previous research [25], possibly due to the overstimulation of ovarian steroidogenesis and decrease of sex hormone-binding globulin blood concentrations mediated by insulin [21]. But there was no significant difference among different weight groups in terms of Gn dose and Gn duration in our study, which means that the high progestin levels in PPOS protocol may partially alleviate the endocrine disorder, and PPOS protocol has potential benefits for overweight patients.

Few studies have shown statistical differences between underweight patients and overweight patients. Some research studies indicated that underweight patients got less embryos [12] as slim patients may face an obstacle of oocyte maturation inhibition. This study found that the underweight patients did not show a poorer ovarian response or a worse embryos outcome compared to normal weight or overweight group, which shows that the PPOS protocol may also have potential benefits for underweight patients.

Since all the embryos were frozen in this protocol and patients should perform the embryo transfer at least one month later, some patients may take much longer time, and only part of these patients have completed the FET process, so the FET pregnancy outcome was not included in the current study, which made it hard to draw a conclusion about whether PPOS has affected the final pregnancy outcome. Moreover, it has been recognized that obesity increased the risk of pregnancy complications, even in natural pregnancy [26]; in the PPOS protocol, the FET outcome may not be the best indicators of the effect of BMI. The FET outcome will be studied in our following studies.

In conclusion, BMI showed no impact on the outcomes of the controlled ovarian stimulation in PPOS protocol. This finding has important implications for overweight patients, as it attains the same effect with normal patients and requires no increase in Gn dose and Gn duration. However, our studies were limited by the sample size and difficulties in reviewing all final pregnancy outcomes. Therefore, further prospective studies with larger sample size and tracking of further results of FET outcomes of PPOS patients should be performed.

## Figures and Tables

**Table 1:** Basic characteristics and hormonal profile of different weight patients.

Characteristic	Normal weight (*n* = 418)	Overweight (*n* = 173)	Underweight (*n* = 45)	*P*
Age (years)	36.2 ± 5.1	36.0 ± 5.8	35.7 ± 5.3	0.801
Duration of infertility (years)	6.3 ± 5.1	5.6 ± 5.0	7.7 ± 6.5	0.051
Previous pregnancy (%)	65.1	68.8	62.2	0.595
Previous IVF failures	0.9 ± 1.0	0.9 ± 1.0	1.1 ± 1.0	0.366
Cause of infertility (%)				
Tubal factor	244 (58.3)	97 (56.1)	29 (64.4)	0.145
Endometriosis	20 (4.8)	17 (9.8)	3 (6.7)	
Dysfunction of ovulation	60 (14.4)	32 (18.5)	5 (11.1)	
Male factor	35 (8.4)	9 (5.2)	1 (2.2)	
Combined factor	59 (14.1)	18 (10.4)	7 (15.6)	
Antral follicle counts	7.9 ± 4.6	7.3 ± 3.7	8.0 ± 4.8	0.249
Basal FSH concentration (mIU/mL)	9.6 ± 4.7	9.6 ± 4.7	9.5 ± 4.4	0.993
Basal LH concentration (mIU/mL)	3.9 ± 2.1	3.8 ± 2.0	3.8 ± 1.9	0.967
Basal E2 concentration (pg/ml)	53.1 ± 43.9	55.8 ± 52.5	55.8 ± 44.9	0.785

**Table 2:** The cycle characteristics of controlled ovarian stimulation of different weight patients.

Characteristic	Normal weight (*n* = 418)	Overweight (*n* = 173)	Underweight (*n* = 45)	*P*
Gn dose (IU)	2458 ± 897	2451 ± 810	2695 ± 871	0.207
Gn duration (days)	9.8 ± 2.9	9.8 ± 2.8	9.9 ± 3.2	0.991
>10 mm follicles on HCG day (*n*)	6.6 ± 5.1	6.9 ± 4.8	7.2 ± 4.1	0.573
>14 mm follicles on HCG day (*n*)	3.9 ± 2.8	4.0 ± 2.5	4.0 ± 2.2	0.947
E2 concentration on HCG day (pg/ml)	1452 ± 1026	1611 ± 1031	1409 ± 946	0.196
Endometrium thickness on hCG day (mm)	7.8 ± 1.8	7.7 ± 1.8	8.3 ± 2.4	0.139
Oocytes retrieved (*n*)	4.3 ± 3.5	4.6 ± 3.3	4.6 ± 2.6	0.622
Fertilized eggs (*n*)	2.9 ± 2.7	3.2 ± 2.8	3.0 ± 2.0	0.430
Cleaved embryos (*n*)	2.8 ± 2.6	3.1 ± 2.7	2.9 ± 2.0	0.436
Fertilization rate (%)	67.7	70.3	66.8	0.008
Cleavage rate (%)	96.8	97.0	95.6	0.724
2PN fertilization rate (%)	57.7	58.7	54.6	0.567
2PN cleavage rate (%)	83.8	82.5	80.3	0.517
Cancellation rate of the cycle (%)	21.8	17.3	20.0	0.477
Top quality of embryos of day 3 (*n*)	1.7 ± 1.7	1.8 ± 1.9	1.7 ± 1.4	0.932

## Data Availability

All of the original data in this study are from the Reproductive Medicine Management System of the Reproductive Center of Renmin Hospital of Wuhan University.
